RETRACTED

# Medical Cloud Computing Data Processing to Optimize the Effect of Drugs

**DOI:** 10.1155/2021/5560691

**Published:** 2021-03-19

**Authors:** Fengxia Li, Zhi Qu, Ruiling Li

**Affiliations:** ^1^Huaihe Hospital of Henan University, Kaifeng 475000, China; ^2^School of Nursing and Health, Henan University, Kaifeng 475001, China

## Abstract

In recent years, cloud computing technology is maturing in the process of growing. Hadoop originated from Apache Nutch and is an open-source cloud computing platform. Moreover, the platform is characterized by large scale, virtualization, strong stability, strong versatility, and support for scalability. It is necessary and far-reaching, based on the characteristics of unstructured medical images, to combine content-based medical image retrieval with the Hadoop cloud platform to conduct research. This study combines the impact mechanism of senile dementia vascular endothelial cells with cloud computing to construct a corresponding data retrieval platform of the cloud computing image set. Moreover, this study uses Hadoop's core framework distributed file system HDFS to upload images, store the images in the HDFS and image feature vectors in HBase, and use MapReduce programming mode to perform parallel retrieval, and each of the nodes cooperates with each other. The results show that the proposed method has certain effects and can be applied to medical research.

## 1. Introduction

Alzheimer's disease (AD) is a neurological disease that is insidious and progressive. The patient's brain is diffusely atrophied, the third ventricle and lateral ventricles are significantly enlarged, and the sea brain is obviously atrophied, and these changes are aggravated with age, which aggravates the patient's condition. Moreover, patients often have memory loss, cognitive dysfunction, behavioral changes, and other symptoms, which cause a greater burden on the patient's family and society [1].

According to statistics, there are about 3 million to 4 million patients with dementia in China. The Beijing Geriatrics Medical Research Center survey of 2788 elderly people over 60 years old in Beijing found that the prevalence of Alzheimer's disease was 7.5%, and the ratio of male-to-female prevalence was 1 : 2. In the survey of elderly people over 75 years old in Guangzhou urban area, the prevalence of AD was 7.49%, and the incidence rate was 45%–80% among 80–85 year olds. According to reports, in 1997, 4 million people in the United States suffered from this disease, ranking fourth among death factors. As the social population ages, the number of patients with AD has risen sharply. Due to the unclear etiology and pathogenesis of the disease, there is no effective prevention and treatment method, which has caused a huge burden on families and society. Studying the etiology, pathogenesis, and prevention of Alzheimer's disease has become an important task in the medical community [2].

RETRACTED

The pathogenesis of AD is related to many factors, and many doctrines have been formed for a long time. The main doctrines are the tau protein theory and the A13 theory. The tau protein theory suggests that abnormal phosphorylation of tau in neuronal cells causes neurofibrillary tangles (NFT) and further causes cytoskeletal rupture, loss of neurons, and synapses, and ultimately brain atrophy. The A13 theory has been proposed for more than ten years [3]. This theory holds that the imbalance between the production and clearance of A6 in the brain tissue is the initial cause of AD. Selkoe [4], on the theory of AD, still believes that the formation and clearance of p-amyloid-protein (Ap) is an early process and central link in the pathogenesis of AD. Genes such as APP (B-amyloid precursor protein) and presenilin are involved in the formation of A13, and clearance of A13 is associated with the inflammatory response. Now, the treatment based on this hypothesis has entered the human experiment stage.

The key question to explore the relationship between immune cells and the formation and clearance of AB is whether immune cells can cross the blood-brain barrier (BBB). Foreign scholars have different views on this issue. Because of the existence of the blood-brain barrier, people have always believed that the brain is an immune exemption organ. However, as research progresses, people gradually realize that the immune exemption of the brain is relative. In the course of a nervous system disease, damage to the blood-brain barrier or activation of peripheral immune cells can cause immune cells to enter the brain and initiate an immune response in the brain. The most critical structure of the blood-brain barrier is the tight junction of brain microvascular endothelial cells [5], also known as zonula occludens. It blocks the intercellular space at the top of the cell and blocks extracellular macromolecular material from entering the tissue through the intercellular space.

It has been suggested that peripheral immune cells of AD patients cannot pass through the BBB because the cell adhesion molecules ICAM-1, VCAM-1, E-selectin, etc., which were previously considered to be most important, were not found on the brain capillary endothelial cells of AD patients. However, studies have shown that AB can increase mononuclear cells through the BBB in vitro model [6]. In order to study whether peripheral blood immune cells of AD patients can cross the blood-brain barrier (BBB) and further study its mechanism, based on the detection of the distribution of peripheral blood immune cell subsets in AD patients, we investigated its ability to cross the in vitro model of the blood-brain barrier and observed changes in tight junction proteins and cytoskeleton between cerebrovascular endothelial cells when interacting with lymphocytes.

RETRACTED

The purpose of this study was to investigate the ability of peripheral blood immune cells in AD patients to cross the blood-brain barrier. Moreover, on this basis, this study used gene chips to search for differentially expressed genes in peripheral blood T lymphocytes of AD patients to study their role in peripheral blood T lymphocytes crossing the blood-brain barrier in AD patients.

## 2. Related Work

The mechanism of content-based image retrieval technology is to measure the similarity between images by calculating the distance between the image to be retrieved and the image in the image database according to some visual features of the image, such as color, shape, texture, and gradient features, and then use the distance as the basis of similarity for matching retrieval [7]. This method makes up for the shortcomings of text-based retrieval technology that is not objective. Content-based image retrieval technology extracts content features directly from the image itself to ensure the objectivity and accuracy of content-based image retrieval technology. This method breaks the limitations of text-based retrieval technology and achieves accurate extraction of image features, making the retrieved similar images closer to ideal retrieval results.

Since the 1990s, content-based medical image retrieval technology has been analyzed and studied at home and abroad, and progress has been made. In recent years, scholars have developed different medical image retrieval systems for different medical tasks not only for single-source medical images, for example, for pathology and imaging images, but also for a variety of medical images that are derived from multiple sources and have implemented retrieval systems.

Wang [8] and his students studied content-based medical image retrieval, and they used brain MR images as research objects. The main extraction method is based on the DT-CWT and GGD models, and they used the Kullback–Leibler distance of the chain rule to measure the similarity to perform feature matching. Zou [9] and others also studied content-based medical image retrieval, which mainly analyzes and proposes a retrieval method that combines wavelet transform and contour features, and proved the effectiveness of the method. Lu et al. [10] first used the neural network to realize segmentation of brain MR images, then extracted features such as shape, texture, image moment, and histogram, and finally realized similarity matching image retrieval. Kapila et al. [11] introduced a new idea of adopting the dual-density dual-tree complex wavelet in the process of medical image texture extraction and introduced the support vector machine active learning algorithm in the retrieval system. Studies have shown that the method is feasible and has great advantages.

RETRACTED

Zhang et al. [12] analyzed the research situation of the content-based medical image retrieval system. The results show that most of the current research studies focus on theory, and the application of content-based medical image retrieval technology to clinical is still very few. Qin et al. [13] developed a high-resolution lung CT image as a research object and developed an automatic search and selection engine search tool ASSERT (Automated Search and Selection Engine with Retrieval Tools). It can use the corresponding algorithm to extract the feature vector unique to the disease image for the difference of lung diseases. First, the doctor submits the image to be retrieved, then judges the category of the disease to which it belongs to and extracts its feature vector, and finally finds a similar image in the database. ASSERT is one of the few clinically based content-based medical image retrieval systems. By testing 11 volunteers, it finally showed that when using ASSERT to assist in the diagnosis and treatment of lung diseases, the precision rate increased from 29% to 62%. Hong et al. [14] developed the CT database system, which has a large number of different CT images of lung diseases. This system first obtains texture feature vectors for all medical images in the library and then builds an image texture feature library. Therefore, when the user needs to find an image, it is convenient and quick to find the desired medical image by comparing the image to be retrieved with the image in the image library.

Xia et al., in conjunction with the Massachusetts Institute of Technology [15], developed the VIR Image Engine medical image retrieval system [16]. The search system incorporates color, texture, and shape features and supports extensions. The user can select one or more of them for a single search or multiple searches. For example, after the first search, the weights between the features can be adjusted according to the results, and then the search is taken again to obtain the desired result. Zheng et al. analyzed various modal medical images and developed the CasImage retrieval system. The system acquires approximately 190-dimensional global, local color features and texture features and integrates them into the PACS to achieve a combination of text and content retrieval. MARS is an image retrieval system supported by the University of Illinois to support low-level features, and MARS is the first CBIR system to provide relevant feedback. The system uses the color histogram of HSV space to describe the image color, extracts the roughness, contrast, and directionality of the image to describe the texture, uses image texture segmentation to realize the content description in the image, and groups the images according to the degree of interest. Because the system uses many methods of feature description and similarity measurement, MARS implements a more abundant search function, such as using Boolean expressions for retrieval [17].

RETRACTED

## 3. Depth Map-Based Method

In computer graphics, a depth map refers to an image that stores vertical distance information from various points to viewpoint positions in a three-dimensional scene.  Figure 1 shows a schematic of the depth map. As can be seen from the definition of the depth map, the image contains three-dimensional contour information of objects in the scene. Therefore, the 3D laser scanning point cloud data can be compressed and stored using the depth map. The depth map can be obtained in two ways [18]: one method is to set the projection mode of the camera in a three-dimensional scene to a parallel projection. Then, the result displayed on the screen is the depth map of the three-dimensional scene; another method is to set the projection mode of the camera to a perspective projection and obtain a depth map by storing the depth buffer.

Figure 2 shows a schematic and principle diagram of a virtual structured-light projection system. In a real measurement system based on the structured light projection, the projection of the projector and the camera is a perspective projection. However, in this virtual system, the projection mode of the projector and the camera are set to be in parallel projection, and the geometric relationship between the two can also be accurately set [19]. In the figure, the spatial extent observed by the camera's viewport corresponds to the unit cube, and the coordinates of the object have been normalized into unit cubes by translation and scaling operations.

It can be seen from Figure 2(b) that, for any point *A* on the camera, if no object is placed on the reference plane, its corresponding phase is the phase Φ_*B*_^*r*^ of point *B* on the reference plane. After placing the object, the phase corresponding to point *A* on the camera is the phase Φ_*C*_ of point *C* on the object. From the perspective of the projector, the phase of point *C* on the object is equal to the phase of point *D* on the reference plane and is equal to the phase projected on the projector, that is, Φ=Φ_*C*_=Φ_*D*_^*r*^. Therefore, the phase change corresponding to point *A* after placing the object is

(1) $$\begin{array}{c} △\Phi =\Phi_{C}-\Phi_{B}^{r}=\Phi_{D}^{r}-\Phi_{B}^{r}=\Phi -\Phi_{B}^{r}. \end{array}$$

If it is assumed that the projection fringe used by the projector is changed in the horizontal direction, the projected stripe width is *P*, and the projection angle of the projector with the virtual camera photographing direction is *θ*, the width of the projected stripe on the reference plane is *P*_*r*_=*P*/cos *θ*. Since the projected fringes on the reference plane are evenly distributed, the phase on the reference plane is defined as a function of *θ* and *P*, that is,

(2) $$\begin{array}{c} \Phi^{r}=\frac{2\pi i}{P_{r}}=\frac{2\pi i\;\cos\;\theta }{P}. \end{array}$$

In the formula, *i* is the camera's horizontal orientation pixel index. From formulas (1) and (2), the following formula can be obtained:

(3) $$\begin{array}{c} △\Phi =\Phi -\frac{2\pi i\;\cos\;\theta }{P}=\frac{2\pi △i\;\cos\theta }{P}. \end{array}$$

Since the spatial extent observed by the camera's viewport corresponds to a unit cube, the space length corresponding to each pixel on the camera is 1/*W*, where *W* is the number of pixels in the camera horizontal direction. The spatial coordinates corresponding to a pixel on the camera can be expressed as

(4) $$\begin{array}{c} x^{n}=\frac{i}{W}, \end{array}$$

(5) $$\begin{array}{c} y^{n}=\frac{j}{W}. \end{array}$$

In the formula, *j* is the pixel index of the camera's vertical direction.

RETRACTED

According to the geometric relationship in Figure 3(b), the following formula can be obtained:

(6) $$\begin{array}{c} z^{n}=\frac{△\theta }{\tan\;\theta }. \end{array}$$

Combining equations (3) and (4), the above equation can be expressed as

(7) $$\begin{array}{c} z^{n}=\frac{P△\Phi }{2\pi W\;\sin\;\theta }=\frac{P\left(\Phi -\left(2\pi i\;\cos\theta /P\right)\right)}{2\pi W\;\sin\;\theta }. \end{array}$$

According to the coordinate (*x*^*n*^, *y*^*n*^, *z*^*n*^), the original three-dimensional coordinates are

(8) $$\begin{array}{c} x=x^{n}\times S_{c}+C_{x},\\ y=y^{n}\times S_{c}+C_{y},\\ z=z^{n}\times S_{c}+C_{z}. \end{array}$$

In the formula, *S*_*c*_ is the scaling factor, and (*C*_*x*_, *C*_*y*_, *C*_*z*_) is the coordinate of the center point of the original 3D object.

It can be seen from the above formula that the spatial coordinates of the object can be calculated according to the image taken by the camera.

Liao et al. [20] proposed the concept of progressive point cloud surface, which uses multiple levels of points to represent the surface. The method is based on a moving least squares method and defines projection operations and refinement rules. Among them, the projection operation is used to determine the position of the new insertion point. Moreover, the refinement rule is used to determine the tangential component of the new insertion point. Through these two operations, a given set of base points can be gradually refined into the original point set. The construction process of the progressive point cloud surface is given in the following.

RETRACTED

For an original point set *R*={*r*_*i*_}, a primitive surface *S*_*R*_ can be obtained using the moving least squares method. A base point set *P*_0_ ⊂ *P* can be obtained by removing a part of the original point set. Similarly, the point set corresponds to a surface *S*_*P*_0__, and the surface is not the same as the original surface. In order to reduce the error between the surface corresponding to the base point set and the corresponding surface of the original point set, it can be implemented by inserting a new point into the base point set.

When a new point is inserted into the base point set, a new point set *P*_1_ is formed. Since the position of the new insertion point does not refer to the original point set, *P*_1_⊄*R*. By moving the new insertion point, the error between the corresponding surface of the newly formed point set and the corresponding surface of the original point set can be reduced, that is, *d*(*S*_*P*_1__, *S*_*R*_) < *d*(*S*_*P*_0__, *S*_*R*_).

By repeating the above interpolation operation, a series of point sets *P*_*i*_ with smaller and smaller surface errors corresponding to the original point set are generated. The MLS surface corresponding to this series of point sets is the progressive point set surface. The progressive compression of the point set can be achieved by encoding the compression by inserting the offset of the point in the point set *P*_*i*_.

Based on MLS spherical surfaces, the fitting implementations such as Guennebaud [21] use multiple levels of points to represent surfaces. Compared with the method proposed by Fleishman, this method is more stable at low sampling rate and high curvature.

Although the above method can achieve progressive compression of point cloud data, using MLS fitting for sharp areas can produce a smoothing effect. Therefore, the above method is not ideal for noisy data processing. Moreover, since the MLS calculation is required at the time of decoding, the MLS method decompression is time consuming.

The compression method based on the virtual structured-light projection system encodes the phase using three channels of the color image and realizes compression storage of the three-dimensional contour data using the 24-bit image by projecting the object and acquiring the deformed image highly modulated by the object. The intensity values of the three channels of the projected image used by the algorithm are as follows:

(9) $$\begin{array}{c} I_{r}\left(i,j\right)=127.5+127.5\;\sin\;\phi , \end{array}$$

(10) $$\begin{array}{c} I_{g}\left(i,j\right)=127.5+127.5\;\cos\;\phi , \end{array}$$

(11) $$\begin{array}{c} I_{b}\left(i,j\right)=\frac{\phi -\text{wrap}\left(\phi \right)}{2\pi }\times \Delta s_{b}. \end{array}$$

In the formula, *i* is the pixel index in the horizontal direction, and *j* is the pixel index in the vertical direction. The *ϕ*=2*πi*/*P*, wrap(*ϕ*) function limits *x* to [−*π*, *π*] by adding or subtracting an integer multiple of 2*π*; Δ*s*_*b*_ represents the gamma difference between adjacent ladders of the B channel.

RETRACTED

According to the above formula, the projection phase can be calculated by the following formula:

(12) $$\begin{array}{c} \Phi \left(i,j\right)=\frac{2\pi I_{b}}{\Delta s_{b}}+\arctan\left(\frac{I_{r}-127.5}{I_{g}-127.5}\right). \end{array}$$

The horizontal direction coding curve and projection phase of the algorithm are shown in Figure 3.  Figure 3(a) is a curve in which the intensity values of the three channels of the projected image are changed in the horizontal direction, and Figure 3(b) is a curve in which the projection phase changes in the horizontal direction.

In the composite phase-shift algorithm, the R and G channels are used to calculate the wrap phase, and the B channel is used to assist in dephasing the phase. The two-channel phase-encoding method replaces the R and G channels used to calculate the wrap phase with one channel while keeping the B channel unchanged, thereby realizing the use of two channels of color images to store 3D contour data and further improving the 3D contour data compression ratio. Among them, the intensity value of the R channel in the two-channel phase-encoding method is determined by the following formula:

(13) $$\begin{array}{c} I_{r}\left(i,j\right)=255\frac{\phi +\pi }{2\pi }. \end{array}$$

According to equations (11) and (13), the projection bit can be calculated by

(14) $$\begin{array}{c} \Phi \left(i,j\right)=\frac{2\pi I_{b}}{\Delta s_{b}}+\frac{2\pi I_{r}}{255}-\pi . \end{array}$$

The method of the horizontal direction coding curve and projection phase are shown in Figure 4.  Figure 4(a) is the curve in which the intensity values of projection images R and B are horizontally changed, and Figure 4(b) is the curve in which the projection phase changes in the horizontal direction.

RETRACTED

Compared with the two-channel phase-encoding method, the B channel in the three-channel phase-encoding method remains unchanged, the G channel subdivides each gray step of the B channel, and the R channel subdivides the subdivided G channel. The intensity variation of the G channel and the R channel in the three-channel phase-encoding method is determined by the following equation:

(15) $$\begin{array}{c} I_{g}\left(i,j\right)=\frac{\phi T-\text{wrap}\left(\phi T\right)}{2\pi }\times \Delta s_{g},\\ I_{r}\left(i,j\right)=255\frac{\left[\text{wrap}\left(\phi T\right)+\pi \right]}{2\pi }. \end{array}$$

In the formula, *T*  represents the number of copies of each step of the G channel to the B channel, and Δ*s*_*g*_ represents the difference in intensity between adjacent steps in the G channel.

The projection phase can be calculated by the following formula:

(16) $$\begin{array}{c} \Phi \left(i,j\right)=\frac{2\pi I_{b}}{\Delta s_{b}}+\frac{\varphi \left(i,j\right)}{T}+\frac{2\pi I_{g}}{T\Delta s_{g}}. \end{array}$$

In the above formula, *φ* can be calculated by the following formula:

(17) $$\begin{array}{c} \varphi \left(i,j\right)=\frac{2\pi I_{r}}{255}-\pi . \end{array}$$

The method of the horizontal direction coding curve and projection phase are shown in Figure 5.  Figure 5(a) is the curve in which the intensity value of the three channels of the projected image is horizontally changed, and Figure 5(b) is the curve in which the projection phase changes in the horizontal direction.

## 4. Gray Value Encoding Method

Compared with the composite phase-shift algorithm, the two-channel phase-encoding method reduces the number of image bits used to store point cloud data but still requires two channels (16 bits) of the color image. Therefore, in order to further reduce the number of image bits required to store 3D laser scanning point cloud data, this paper proposes a gray value encoding method.

Since the resolutions of the virtual projector and the virtual camera are the same and the fringe image for projection is changed in the horizontal direction, for the case where the horizontal resolution of the virtual camera is *W* (that is, the horizontal resolution of the resulting image), it is only necessary to encode the *W* values in the horizontal direction so that the values along the vertical direction can be kept constant to ensure the uniqueness of the information to be encoded in the horizontal direction. For a commonly used 8-bit grayscale image, the gray value is between [0,255], and there are 256 gray levels. For a *k*-bit grayscale image, the gray value is between [0, 2^*k*^ − 1], and there are 2^*k*^ gray levels. Therefore, we can achieve correct decoding of the captured image by encoding some or all of the gray values in the gray value [0, 2^*k*^ − 1] of the *k*-bit image.

RETRACTED

According to the above ideas, this paper proposes a gray value encoding method. First, the number of image bits used to encode the gray value is determined according to the horizontal direction resolution *W* of the virtual camera. Then, the *N* gradation values in [0, *N* − 1] are encoded according to the index value of the pixel and stored as a two-dimensional image. In order to ensure the uniqueness of the encoded information in the horizontal direction, the number of gray values to be encoded is equal to the horizontal resolution of the virtual camera, that is, *N*=*W*. When *W* ≤ 256, the 8-bit grayscale image has a total of 256 gray levels, which can satisfy the encoding of *W* values. Therefore, *N* gradation values in [0, *N* − 1]*g* can be encoded as a single 8-bit grayscale image based on the index value of the pixel. When *W* > 256, at least *k*=[log  *W*]-bit image is required to encode the *W* values. Commonly used grayscale images are 8 bits, 24 bits, and 32 bits. If the encoding result of the gray value is stored using the *k*-bit in the 24-bit image, the storage space is wasted, and the encoded image size is increased. In order to reduce the size of the encoded image, it is necessary to use as few image bits as possible to store the encoded result. Therefore, this paper uses a single 8-bit grayscale image combined with *M*=*k* − 8=[log_2_  *W*] − 8,  (*W* > 256)-frame 1-bit binary image to store the encoded result. The single 8-bit grayscale image and a 1-bit binary image can be obtained by the following formula.

The single 8-bit grayscale image can be represented as

(18) $$\begin{array}{c} I_{\text{gray}}\left(i,j\right)=\mathrm{mod}\left[G\left(i,j\right),256\right]. \end{array}$$

In the formula, *i* ∈ [0, *W* − 1], *j* ∈ [0, *H* − 1], *H* is the resolution of the camera in the vertical direction, *I*_gray_(*i*, *j*) is the gray value after the pixel whose index value is (*i*, *j*) is encoded, mod(*a*, *b*) represents the remainder operation, and *G*(*i*, *j*) is the gray value to be encoded at the pixel point whose index value is (*i*, *j*). In order to ensure that the gray value to be encoded is within [0, *N* − 1] and the coding result changes simply, the index value of the horizontal-direction pixel is used to assign it, that is, *G*(*i*, *j*)=*i*. It increases in the horizontal direction and remains unchanged in the vertical direction.

When the camera horizontal resolution is greater than 256 pixels, that is, *W* > 256, in addition to storing the gray value code as a single 8-bit gray image according to formula (18), it is also necessary to store the grayscale value encoding result using an *M*-frame 1-bit binary image. The binary image can be expressed as

(19) $$\begin{array}{c} I_{{\text{binary}}_{m}}\left(i,j\right)=\mathrm{mod}\left\{\left\lfloor \frac{\left[G\left(i,j\right)-I_{\text{gray}}\left(i,j\right)\right]}{2^{m+7}}\right\rfloor ,2\right\},\;m\in \left[1,M\right]. \end{array}$$

In the formula, *m* is the index of the binary image, and *I*_binary_*m*__(*i*, *j*) is the gray value after the pixel with the index value *h* on the *m*-th binary image is encoded.

RETRACTED

After encoding by the above formula, the *N* gray values in [0, *N* − 1] are encoded into a single 8-bit grayscale image or a single 8-bit grayscale image and an *M*-frame 1-bit binary image. Since the integer is used for encoding the gray value, the quantization error caused by the direct conversion of the floating point data to the integer data when the phase (*ϕ*(*i*, *j*)=2*πi*/*P*, where *P* is the number of pixels in the horizontal direction of the stripe) is encoded is avoided. The method proposed in this paper stores the encoding result of the gray value using as few image bits as possible, and the encoded gray image and binary image change are simple, thus further reducing the size of the encoded image.

When the camera's horizontal resolution is less than or equal to 256 pixels, that is, *W* ≤ 256, the encoded gray value is

(20) $$\begin{array}{c} G\left(i,j\right)=I_{\text{gray}}\left(i,j\right). \end{array}$$

When the camera's horizontal resolution is greater than 256 pixels, that is, *W* > 256, the encoded gray value is

(21) $$\begin{array}{c} G\left(i,j\right)=I_{\text{gray}}\left(i,j\right)+\sum_{m=1}^{M}2^{m+7}I_{{\text{binary}}_{m}}\left(i,j\right). \end{array}$$

Since the phase information in the coded image can be expressed as *h* (the method proposed in this paper is to encode *m* gray values, that is, equivalent to *n*) and encode the gray value, the phase corresponding to the gray value is as follows: since the phase information in the coded image can be expressed as *ϕ*(*i*, *j*)=2*πi*/*P* (the method proposed in this paper encodes *N*=*W* gradation values, that is, equivalent to *P*=*W*) and the gradation value of the code is *G*(*i*, *j*)=*i*, the phase corresponding to the gray value is

(22) $$\begin{array}{c} \Phi \left(i,j\right)=\frac{2\pi G\left(i,j\right)}{W}. \end{array}$$

The phase obtained here is between 0 and 2*π*, and there is no discontinuity of the 2*π* phase, thus avoiding the phase unwrapping operation.  Figure 6 is a graph showing the variation of the encoding and decoding results of the proposed method in the horizontal direction in the case where the camera has a horizontal resolution of 1024 pixels.  Figure 6(a) is a gray value of the encoded grayscale image in the horizontal direction; Figure 6(b) is a gray value of the first encoded binary image in the horizontal direction; Figure 6(c) is a gray value of the second encoded binary image in the horizontal direction; Figure 6(d) is the gray value encoded in the horizontal direction; and Figure 6(e) is a phase corresponding to the gray value encoded in the horizontal direction.

RETRACTED

The coding result is projected onto the three-dimensional point cloud data as a projection image, and the projection image is deformed after being highly modulated by the data. At this time, the grayscale image *I*_gray_′ or the grayscale image *I*_gray_′ and the binary image *I*_binary_*m*__′ which are deformed using the data captured by the virtual camera include the three-dimensional point cloud information. The gray value *G*′ modulated by the point cloud data can be obtained by replacing *I*_gray_ in formula (20) with *I*_gray_′ or by replacing *I*_gray_ and *I*_binary_*m*__ in the formula with *I*_gray_′ and *I*_binary_*m*__′. By substituting the gradation value, a phase Φ′ containing the three-dimensional point cloud information can be obtained, and then the original coordinates of the point cloud can be obtained based on the obtained phase Φ′.

All of the above operations are written in OpenGL Shading Language (GLSL), and the real-time reconstruction and display of the 3D point cloud data can be realized by using the parallel processing capability of the GPU.

In order to verify the effectiveness of the proposed method, we experimented with simple and complex models and compared it with other methods. In the following experiment, the virtual camera in the virtual structured-light projection system has a resolution of 512 × 512 pixels, and the other method has a stripe width *P* of 58 pixels, and the angle *θ* between the projection direction and the camera shooting direction is 30°. In order to obtain high data compression ratio while ensuring high reconstruction accuracy, this paper saves the final result as a small, lossless PNG image format.

We first performed a reconstruction experiment on the computer-generated *XYZ* format and a simple ideal unit hemisphere (including 197,824 points). The experimental results are shown in Figure 7. The error results of the reconstruction result and the ideal unit hemisphere are shown in Figure 8. Figure 7(a) shows the original ideal unit hemisphere point cloud data, and Figures 7(b) and 7(h) show the Holoimage method storage and reconstruction results. Figures 8(a) and 8(f) are the error results of the reconstructed model and the ideal unit hemisphere cross-section error and the error diagram of the reconstructed model and the ideal unit hemisphere, respectively. It can be seen from the figure that the surface of the Holoimage method is very smooth, and the error with the ideal unit hemisphere is small, and the root mean square error is about 0.34%. For the Holoimage method, the projection map is subjected to texture interpolation filtering processing during its projection, and the error caused by texture interpolation is filtered by the median filter during the reconstruction calculation, so the restoration result is very smooth. The results of the two-channel phase-encoding method are shown in Figures 7(c), 7(i), 7(b), and 7(g). It can be seen from the figures that the method achieves the restoration of the model as a whole, but there are stepped stripes on the surface of the reduction result, and the error is larger than the Holoimage method, and the root mean square error is about 0.39%. The results of the Bayer dithering method are shown in Figures 7(d), 7(j), 8(c), and 8(h). The results of the Floyd–Steinberg dithering method are shown in Figures 7(e), 7(k), 8(d), and 8(i). The storage results are shown in Figures 7(f) and 7(g). The reduction results of the proposed method are shown in Figure 7(l), and the error results are shown in Figures 8(e) and 8(j). It can be seen from the figures that the method of reducing the method is similar to the two-channel method, and the root mean square error is about 0.36%. The stepped streaks on the surface of the reduction result are mainly due to the same phase value. When the angle between the projector and the camera is greater than zero degrees, one pixel on the projected image is wider than one pixel on the reference plane so that the same phase appears, and finally, the stepped stripe is generated.

RETRACTED

## 5. Image Processing Method Based on the Composite Dithering Algorithm

Due to the limited color range of early displays, screens in mobile phones, and some low-end display devices, it is difficult to represent rich natural images. Therefore, in order to use limited color to represent a wider range of colors, dithering method has emerged. The method converts a continuous tone image into a binary image by a quantization technique, that is, converts the high image into a low image. Since the human eye has a low-pass characteristic, the halftone image looks similar to the original continuous tone image when viewed at a certain distance. The dithering method can be divided into random dithering, ordered dithering, and error diffusion dithering. This article only introduces two common methods of dithering.

Bayer dithering is a type of ordered dithering. The method quantizes the image using a threshold matrix. When the gray value of the current pixel of the image to be processed is greater than the corresponding point gray value in the threshold matrix, the gray value of the point in the result image is assigned a value of 1. When the gray value of the current pixel of the image to be processed is smaller than the corresponding point gray value in the threshold matrix, the gray value of the point in the result image is assigned a value of 0. Bayer found that if the size of the threshold matrix is 2^*n*^ (*n* is an integer), the optimal threshold matrix can be obtained. Among them, the minimum 2 × 2 threshold matrix is

(23) $$\begin{array}{c} M_{1}=\left[\begin{array}{cc} 0 & 2\\ 3 & 1 \end{array}\right]. \end{array}$$

The larger matrix can be obtained by the following formula:

(24) $$\begin{array}{c} M_{n+1}=\left[\begin{array}{cc} 4M_{n} & 4M_{n}+2U_{n}\\ 4M_{n}+3U_{n} & 4M_{n}+U_{n} \end{array}\right]. \end{array}$$

In the formula, *U*_*n*_ is an *n*-dimensional unit matrix. The larger the threshold matrix, the more the corresponding threshold, the smaller the quantization error in the coding result, and the less obvious the artificial trace.

The advantage of Bayer dithering is that it is simple to compute and can be processed in parallel. However, the threshold matrix used by the algorithm will bring a block quantization error to the coding result, resulting in a large error in decoding.

We assume that the original continuous tone image is *f*, the highest gray level is *g*, and the image obtained by the error diffusion dithering of the continuous tone image is *b*. The processing block diagram of the error diffusion dithering algorithm is shown in Figure 9. In the figure, *u*(*i*, *j*) is the intermediate result of the dithering calculation, which is expressed as follows:

(25) $$\begin{array}{c} u\left(i,j\right)=f\left(i,j\right)+\sum_{k,l}h\left(k,l\right)e\left(i-k,j-l\right). \end{array}$$

In the formula, *h*(*k*, *l*) is the error diffusion kernel coefficient, and *e*(*i*, *j*) is the quantization error. It can be seen from the formula that the error of the left and the top of the current point is added to the current point by a certain ratio, that is, the error of the left and the upper is spread to the current point. The error diffusion kernel coefficient satisfies the following conditions:

(26) $$\begin{array}{c} h\left(k,l\right)\geq 0,\\ \sum_{k,l}h\left(k,l\right)=1. \end{array}$$

The error diffusion kernel of the Floyd–Steinberg dithering algorithm is as follows:

(27) $$\begin{array}{c} \begin{array}{ccc} & * & \frac{7}{16}\\ \frac{3}{16} & \frac{5}{16} & \frac{1}{16} \end{array}. \end{array}$$

In the algorithm, the blank represents the pixel that has been processed, the asterisk represents the pixel to be processed, and the four fractions represent the proportion of the error spread to the adjacent pixel.

RETRACTED

The intermediate result *u*(*i*, *j*) of the dithering calculation is quantized to obtain the dithering result *b*(*i*, *j*). The quantization function is as follows:

(28) $$\begin{array}{c} Q\left(u\right)=\left\{\begin{array}{cc} 1, & u\geq \frac{g}{2},\\ 0, & u<\frac{g}{2}. \end{array}\right. \end{array}$$

The quantization error of the current point is calculated according to the intermediate result of the dithering calculation and the quantization result, and the formula is as follows:

(29) $$\begin{array}{c} e\left(i,j\right)=u\left(i,j\right)-b\left(i,j\right). \end{array}$$

The Floyd–Steinberg dithering algorithm reduces the cumulative error of the image and reduces the artifacts in the resulting image by spreading the quantization error to adjacent pixels. Unlike the Bayer dithering method that can be computed in parallel, this method requires pixel-by-pixel calculations, so the computation time is longer than the Bayer dithering algorithm.

By using the characteristics that the dithering method can reduce the number of image bits, Karpinsky et al. proposed a method of using 3 bits to represent the 3D laser scanning point cloud data. The color image in which the three-dimensional laser scanning point cloud data are stored in the method is obtained by using a virtual structured-light projection system. Among them, the gray values of the three channels R, G, and B of the projected image used by the virtual structured-light projection system are determined by the following formula:

(30) $$\begin{array}{c} I_{r}\left(i,j\right)=127.5+127.5\;\sin\left(\frac{2\pi i}{P}\right), \end{array}$$

(31) $$\begin{array}{c} I_{g}\left(i,j\right)=127.5+127.5\;\cos\left(\frac{2\pi i}{P}\right), \end{array}$$

(32) $$\begin{array}{c} I_{b}\left(i,j\right)=S\cdot Fl\left(\frac{i}{P}\right)+\frac{S}{2}+\frac{\left(S-2\right)}{2}\cdot \cos\left[\frac{2\pi \cdot \text{Mod}\left(i/P\right)}{P_{1}}\right]. \end{array}$$

In the formula, *i* and *j* are the horizontal and vertical index of the pixel in the image, respectively; *P* is the number of pixels occupied by each stripe; *P*_1_=*P*/(*K*+0.5) is the number of pixels occupied by the stripes in the trapezoidal curve, where *K* is an integer; *S* is the gray level height in the trapezoidal curve; Mod(*a*, *b*) is the remainder operation; and *Fl*(*x*) is the downward rounding operation.

Before the point cloud data are restored, the low-level image obtained by the method needs to be processed to be restored to the original image as much as possible. For the dithering method, it can be processed using a low-pass filter. The obtained low-order image is processed using a Gaussian filter, and the processing result is as shown in Figure 10.  Figure 10(a) is an image in which the unit hemispherical point cloud data are stored, and Figures 10(b) and 10(c) are Figure 10(a) results after Bayer dithering and Floyd–Steinberg dithering, respectively. As can be seen from the figures, the Bayer dithering method has obvious artifacts. Figures 10(d) and 10(e) show the results of Gaussian filter processing in Figures 10(b) and 10(c), respectively. It can be seen from the figures that Bayer dithering and Floyd–Steinberg dithering results are blurred after Gaussian processing. Compared with the Bayer dithering method, the Floyd–Steinberg dithering method spreads the error to adjacent pixels, so the result of the method is Gaussian processing and is closer to the original image, and its error is lower.

RETRACTED

For the Bayer dithering method, the processing result is small, the storage space is small, and the compression ratio is high, but the reconstruction error is large. For the Floyd–Steinberg dithering method, although the reconstruction error is low, the processing result is irregular, the required storage space is large, and the compression ratio is low. In this paper, the Bayer dithering method and the advantages of the Floyd–Steinberg dithering method are combined to propose a composite dithering method. This paper uses different dithering methods for storing different channels of 3D laser scanning point cloud data images, which maintain a low reconstruction error while ensuring a high data compression ratio.

The trapezoidal curve of the cosine variation in formula (32) makes the projection pattern change complicated and causes the image storing the point cloud data to occupy a large storage space, thereby reducing the data compression ratio. In order to reduce the size of the resulting image, the cosine component in equation (32) is removed, and a simpler trapezoidal curve is used. The specific formula is as follows:

(33) $$\begin{array}{c} I_{b}\left(i,j\right)=S\cdot Fl\left(\frac{i}{2}+\frac{1}{2}\right). \end{array}$$

According to equations (30), (31), and (33), the projection phase can be calculated by the following formula:

(34) $$\begin{array}{c} \Phi \left(i,j\right)=2\pi \times Fl\left(\frac{I_{b}}{S}\right)+\phi =2\pi \times Fl\left(\frac{I_{b}}{S}\right)\\ =\text{arcta}\left(\frac{I_{r}-127.5}{I_{g}-127.5}\right). \end{array}$$

In the formula, *ϕ* is the wrapping phase.

RETRACTED

The variation curve of the three channels of the projected image along the horizontal direction and the parcel phase in the projected image are as shown in Figure 11. Among them, the curves corresponding to formulas (30), (31), and (33) are as shown in Figure 11(a), and the wrap phase in formula (34) is as shown in Figure 11(b). From equation (34) and Figure 11, it can be seen that the R and G channels of the projected texture are used to calculate the wrap phase, and the B channel is used to assist in dephasing the phase. When the error of the B channel is less than the height *S* of the step curve, the resulting phase error is 2*π*, which can be filtered by median filtering. Therefore, the channel can be processed with a Bayer dithering method with larger errors and less results. The accuracy of the R and G channels will affect the accuracy of the wrapped phase in equation (34). In order to maintain high reconstruction accuracy while reducing the data size, the Floyd–Steinberg dithering method with low reconstruction error is used for the R channel, and the Bayer dithering method with smaller processing result is used for the G channel. Through the above strategy, the algorithm can maintain a low reconstruction error while achieving a high data compression ratio.

In order to verify the effectiveness of the proposed algorithm, the proposed algorithm is applied to the computer-generated ideal unit sphere and the rabbit model of Stanford University. The image used in the test has a resolution of 512 × 512 pixels, the stripe width of one cycle is 54 pixels, and the projection direction of the projector is 30° from the camera shooting direction. In order to reduce the space occupied by the coding result and ensure high reconstruction accuracy, the coding result is stored here as a small, lossless PNG format.

The experimental results of the unit hemisphere are shown in Figure 12. Figure 12(a) shows the Holoimage result, and the reconstruction result is shown in Figure 12(e). For Figures 12(b)–12(d) using the dithering method, low-pass filtering is required before reconstruction. This paper uses a Gaussian filter with a parameter width of 7 × 7 and a standard deviation of 7/3. The result of the reconstruction of the dithering result after Gaussian filtering is shown in Figures 12(f)–12(h). The result of comparing the cross section of the reconstruction result with the cross section of the ideal unit hemisphere is shown in Figure 13. It can be seen from the figure that the Holoimage method reconstructs the smoothest surface and has a root mean square error of about 0.32%. The reconstruction results of Bayer's dithering method have obvious random noise on the surface, while the Floyd–Steinberg dithering method has random noise on the surface, but the reconstruction result is better than that of the Bayer dithering method. The root mean square errors of the two methods were 0.62% and 0.39%, respectively. The error of most points in the composite dithering method proposed in this paper is close to the Floyd–Steinberg dithering method, and only the individual point error is close to the Bayer dithering method. The method has a root mean square error of approximately 0.43%, which is between the Bayer and Floyd–Steinberg dithering methods and guarantees high reconstruction accuracy.

RETRACTED

## 6. Vascular Endothelial Cell Research System Based on Cloud Computing for Alzheimer's Disease Patients

The research goal of this project is to realize the medical image recognition system in the cloud computing environment based on the Hadoop platform. Users can quickly and accurately retrieve a large number of medical images on the platform and quickly find the files combined with vascular endothelial cells to make corresponding judgments, as shown in Figure 14.

The storage module is mainly responsible for storing images, image feature vectors, and index data and is designed as a distributed file system HDFS and a distributed database (HBase). Medical images and index data are stored directly on the HDFS, and image feature vector data are stored in HBase. It can also be seen from Figure 14 that HBase is based on the HDFS.

The main task of the feature extraction module is to upload medical images to the HDFS. Then, a MapReduce job task is started, and the feature extraction algorithm is used to extract the features and store the feature vectors in HBase. Since the number of images is large, the extraction time of image features will be longer. Therefore, in this process, one also needs to call a MapReduce job to speed up the implementation.

The main function of the index module is to speed up the image retrieval speed to index the database of image feature vectors. This article uses LIRE to extract features to build an index. The process of creating an index is relatively time consuming. To reduce the loss, we need to call MapReduce job to quickly complete the indexing process.

The query module is mainly composed of two parts: a querier and a user interface, in which the user interacts with the entire system through the interface. After the user uploads the image to be retrieved, the system passes it to the querier, and the querier returns the retrieval result to the user through the interface. The style of the interface design should be consistent with the use of the system itself so that it is simple and easy to use, and the overall structure is harmonious and beautiful.

RETRACTED

Stored procedures are the premise and basis for retrieval. When the number of images is large, the extraction time of image features will be longer. This article needs to call a MapReduce job to implement it; its feature extraction and storage framework are shown in Figure 15.

The experimental operating system is Ubuntu 14.04 64-bit operating system, Hadoop-0.20.0 platform is conFig.d, the development environment is Eclipse, and a distributed system consisting of four nodes is built. The processor of the computer is Intel(R) Core(TM) i7-3770 CPU @ 3.40 GH, the memory is 8 GB, and the hard disk is 1 TB. The experimental environment requires four machines: one computer is treated as a NameNode node and the other three are treated as DataNode nodes. In the experiment, we first studied the changes of tight junction protein ZO-1 and cytoskeletal protein F-actin after the interaction of brain microvascular endothelial cells with T lymphocytes.

After 20 hours of interaction between the HBMEC monolayer and peripheral blood T lymphocytes of AD patients, the continuity of tight junction protein ZO-1 disappeared, showing punctate fluorescence, indicating the disappearance of tight junction protein ZO-1 and the destruction of tight junctions. However, after the HBMEC monolayer interacted with normal elderly T lymphocytes for 20 hr, the expression of the blood-brain barrier tight junction protein ZO-1 was slightly discontinuous but still showed a substantially continuous line shape, as shown in Figure 16.

In the absence of lymphocyte action, that is, under normal conditions, ZO-1 is continuously linearly fluorescent at the tight junction of the blood-brain barrier. After 4T-CEM interacted with HBMEC for 4 hr, the distribution of tight junction protein ZO-1 was slightly discontinuous. When 4T-CEM interacted with HBMEC for 8 hr, the ZO-1 discontinuity was aggravated. When 4T-CEM interacted with HBMEC for 20 hr, the continuity of ZO-1 was completely destroyed and spotted, indicating the disappearance of tight junction proteins and complete destruction of tight junctions. It is suggested that the decrease in the expression of tight junction proteins is related to the action time of lymphocytes. This is consistent with the inability of lymphocytes to cross the BBB in vitro model within 12 hours of the preexperiment, as shown in Figure 17.

After HBMEC interacted with peripheral blood T lymphocytes of AD patients for 20 hours, the HBMEC of the cytoskeletal protein F-actin interacted with normal elderly T lymphocytes became thinner and sparsely distributed, as shown in Figure 18.

In Figure 19, after 4 hours of interaction, the cytoskeletal protein F-actin of HBMEC cells became thin and disordered. At 8 hours of interaction, F-actin became uneven in thickness, and the length was different, but the cell edge was clear. After 20 hours of interaction, F-actin became more uneven, the length was different, the number was reduced, and the cell edge was unclear.

RETRACTED

Based on the analysis of the cloud computing platform, this paper firstly found that the ability of peripheral blood T lymphocytes to cross the blood-brain barrier in AD patients was significantly increased on the basis of analyzing the changes of peripheral blood immune cell subsets in AD patients. At the same time, it was found that peripheral blood T lymphocytes of AD patients can cause tight junctional destruction and decreased expression of endothelial cytoskeletal protein F-actin when exposed to microvascular endothelial cells of the blood-brain barrier. Moreover, T lymphocytes cause rearrangement of endothelial cells ZO-1 and actin filaments. As the interaction time between the two cells increases, the disruption of cytoskeletal rearrangement and tight junctions is aggravated. It is directly suggested that T cells may cross the blood-brain barrier by causing cytoskeletal changes and disrupting tight junctions and participate in the pathogenesis of AD. As for what kind of molecules of T cells in AD patients act on brain microvascular endothelial cells, it is a problem we need to study further.

## 7. Conclusion

Aiming at the problem that the Bayer dithering method has a small storage space, but the reconstruction error is high, and the Floyd–Steinberg dithering method has low error, but the storage space required for processing results is large, this paper proposes a composite dithering method. By processing the image storing the 3D laser scanning point cloud data, this study reduces the size of the stored 3D laser scanning point cloud data image as much as possible while maintaining low reconstruction error.

This paper combines the custom LIRE and Hadoop platform to achieve a large number of medical images' retrieval and uses Hadoop's core framework distributed file system HDFS to upload images first and store the images in the HDFS and image feature vectors in HBase. Moreover, this paper uses the MapReduce programming mode for parallel retrieval, and each node cooperates with each other. In addition, this paper designs and implements a more efficient content-based medical image retrieval system under the Hadoop platform. The final experimental results show that the system can effectively improve the accuracy and retrieval efficiency of a large number of medical images and can meet the clinical needs.

RETRACTED

In this paper, for the purpose of remote 3D visualization of laser scanning point cloud data, some research works have been done on the organization, compression, and scheduling of point cloud data. However, due to factors such as experimental conditions, time constraints, and limited personal research capabilities, some methods in this paper are still insufficient and need to be further optimized.

## Figures and Tables

**Figure 1:** Schematic diagram of the depth map.

**Figure 2:** Virtual structured-light projection system. (a) Schematic diagram. (b) Schematic.

**Figure 3:** Coding curve and projection phase in the horizontal direction of the composite phase-shift algorithm.

**Figure 4:** Coding curve and projection phase in the horizontal direction of the two-channel phase-encoding method.

**Figure 5:** The coding curve and projection phase in the horizontal direction of the three-channel phase-encoding method.

**Figure 6:** The curve of the encoding and decoding results of the proposed method in the horizontal direction.

**Figure 7:** Results of the ideal unit hemisphere experiment in different methods.

**Figure 8:** Comparison of 3D reconstruction results of different methods with the ideal unit hemisphere.

**Figure 9:** Block diagram of error diffusion dithering processing.

**Figure 10:** Image dithering and Gaussian processing results.

**Figure 11:** Coding curve and package phase.

**Figure 12:** Unit hemisphere experiment results.

**Figure 13:** Reconstruction error of the unit hemisphere.

**Figure 14:** Overall structure of the system.

**Figure 15:** Storage architecture diagram.

**Figure 16:** Changes in the blood-brain barrier tight junction protein ZO-1 after the HBMEC monolayer interacted with peripheral blood T lymphocytes in AD patients for 20 hr. The ruler is 20 um. (a) The blood-brain barrier tight junction protein ZO-1 after the HBMEC monolayer interacted with peripheral blood T lymphocytes in AD patients for 20 hr. (b) The blood-brain barrier tight junction protein ZO-1 after the HBMEC monolayer interacted with normal-aged peripheral blood T lymphocytes for 20 hr.

**Figure 17:** Changes in tight junction protein ZO-1 of HBMEC cells interacting with 6T-CEM cells. The ruler is 20 um. (a) ZO-1 of HBMEC that does not interact with 6T-CEM cells. (b) ZO-1 of HBMEC after 4 hours of action with 6T-CEM cells. (c) ZO-1 of HBMEC after 8 hours of action with 6T-CEM cells. (d) ZO-1 of HBMEC after 20 hours of action with 6T-CEM cells.

**Figure 18:** Changes in cytoskeletal protein F-actin after vascular endothelial cells interacted with peripheral blood T lymphocytes in AD patients for 20 hours. The ruler is 20 um. (a) Skeletal protein F-actin of HBMEC cells interacting with peripheral blood T lymphocytes of AD patients for 20 hours. (b) Skeletal protein F-actin of HBMEC cells interacting with peripheral blood T lymphocytes of normal age for 20 hours.

RETRACTED

**Figure 19:** Changes in cytoskeletal protein F-actin when vascular endothelial cells interact with 6T-CEM cells. The ruler is 20 um. (a) F-actin of HBMEC that did not interact with 6T-CEM cells. (b) F-actin after 4 hours of action of HBMEC and 6T-CEM cells. (c) F-actin after 8 hours of action of HBECEC and 6T-CEM cells. (d) F-actin after 20 hours of HBMEC interaction with 6T-CEM cells.

## Data Availability

The data used to support the findings of this study are available from the corresponding author upon request.

## References

[1] Jack C. R., Bennett D. A., Blennow K. (2018). NIA-AA research framework: toward a biological definition of Alzheimer’s disease. *Alzheimer’s & Dementia*.

[2] Sims R., Lee S. J. V. D., Naj A. C. (2017). Rare coding variants in PLCG2, ABI3, and TREM2 implicate microglial-mediated innate immunity in Alzheimer’s disease. *Nature Genetics*.

[3] Nakamura A., Kaneko N., Villemagne V. L. (2018). High performance plasma amyloid-*β* biomarkers for Alzheimer’s disease. *Nature*.

[4] Rathore S., Habes M., Iftikhar M. A. (2017). A review on neuroimaging-based classification studies and associated feature extraction methods for Alzheimer’s disease and its prodromal stages. *NeuroImage*.

[5] Espuny-Camacho I., Arranz A. M., Fiers M. (2017). Hallmarks of Alzheimer’s disease in stem-cell-derived human neurons transplanted into mouse brain. *Neuron*.

[6] Sasaguri H., Nilsson P., Hashimoto S. (2017). APP mouse models for Alzheimer’s disease preclinical studies. *The EMBO Journal*.

[7] Bachurin S. O., Bovina E. V., Ustyugov A. A. (2017). Drugs in clinical trials for Alzheimer’s disease: the major trends. *Medicinal Research Reviews*.

[8] Wang Y., Miao M., Shen J. (2019). Towards efficient privacy-preserving encrypted image search in cloud computing. *Soft Computing*.

[9] Zou Q., Wang J., Ye J. (2017). Efficient and secure encrypted image search in mobile cloud computing. *Soft Computing*.

[10] Lu W., Varna A. L., Wu M. (2014). Confidentiality-preserving image search: a comparative study between homomorphic encryption and distance-preserving randomization. *IEEE Access*.

[11] Kapila R., Jayalakshmi N., Rao M. S. (2014). A new image search model BY tagging for estimating user search criteria. *International Journal of Innovative Technology and Research*.

[12] Zhang C., Cheng K., Zhu L. (2019). Efficient continuous top-k geo-image search on road network. *Multimedia Tools and Applications*.

RETRACTED

[13] Qin Z., Weng J., Cui Y., Ren K. (2018). Privacy-preserving image processing in the cloud. *IEEE Cloud Computing*.

[14] Hong R., Li L., Cai J. (2017). Coherent semantic-visual indexing for large-scale image retrieval in the cloud. *IEEE Transactions on Image Processing*.

[15] Xia Z., Wang X., Zhang L. (2017). A privacy-preserving and copy-deterrence content-based image retrieval scheme in cloud computing. *IEEE Transactions on Information Forensics & Security*.

[16] Zheng Y., Cui H., Wang C., Zhou J. (2017). Privacy-preserving image denoising from external cloud databases. *IEEE Transactions on Information Forensics and Security*.

[17] Kune R., Konugurthi P. K., Agarwal A., Chillarige R. R., Buyya R. (2017). Xhami-extended HDFS and MapReduce interface for Big Data image processing applications in cloud computing environments. *Software: Practice and Experience*.

[18] Xia Z., Xiong N. N., Vasilakos A. V., Sun X. (2017). EPCBIR: an efficient and privacy-preserving content-based image retrieval scheme in cloud computing. *Information Sciences*.

[19] Liao J., Yang D., Li T., Wang J., Qi Q., Zhu X. (2014). A scalable approach for content based image retrieval in cloud datacenter. *Information Systems Frontiers*.

[20] Liao J., Yang D., Li T., Qi Q., Wang J., Sun H. (2016). Fusion feature for LSH-based image retrieval in a cloud datacenter. *Multimedia Tools and Applications*.

[21] Liu X., Zhang L., Lu K. (2015). A 3D image quality assessment method based on vector information and SVD of quaternion matrix under cloud computing environment. *IEEE Transactions on Cloud Computing*.

